# Correlation between Glucose/C-Peptide Ratio and the Risk of Disease Progression in Diabetic Nephropathy Patients: A Clinical Retrospective Analysis

**DOI:** 10.1155/2022/7406764

**Published:** 2022-03-30

**Authors:** Huomu Tong, Dongying Wang, Miaozhen Fang

**Affiliations:** Department of Endocrinology, Chun'an Branch of Zhejiang Provincial People's Hospital, Hangzhou 311700, Zhejiang Province, China

## Abstract

The aim of this study is to analyze the correlation between the glucose/C-peptide ratio and the risk of disease progression in patients with diabetic nephropathy. Ninety-three patients with diabetic nephropathy, who were treated in the Chun'an Branch of Zhejiang Provincial People's Hospital, China, from January 2016 to January 2019, were recruited as subjects. In accordance with the disease progression, the patients were divided into a progression group (*n* = 59) and a nonprogression group (*n* = 34). Clinical data were compared between the two groups. Pearson's correlation was applied to analyze the correlation of age, postprandial glucose/C-peptide, glycosylated hemoglobin, insulin resistance index, serum cystatin C, uric acid, 24 h urinary albumin excretion rate (24 hUAER), and estimated glomerular filtration rate (eGFR). Univariate and multivariate logistic regression models were utilized to analyze the influencing factors for the risk of disease progression in patients with diabetic nephropathy. The receiver operating characteristic (ROC) curve was employed to assess the predictive value of postprandial glucose/C-peptide on the risk of disease progression in patients with diabetic nephropathy. *Results*. The age differences, postprandial glucose/C-peptide, glycosylated hemoglobin, insulin resistance index, serum cystatin C, uric acid, 24 hUAER, and eGFR were significantly different between the two groups (*P* < 0.05). Pearson's linear correlation analysis exhibited that postprandial glucose/C-peptide, insulin resistance index, serum cystatin C, and uric acid were positively correlated with 24 hUAER (*r* = 0.514, 0.345, 0.311, 0.279, *P* < 0.05). Age, postprandial glucose/C-peptide, insulin resistance index, serum cystatin C, and uric acid were negatively correlated with eGFR (*r* = −0.210, −0.610, −0.351, −0.347, and −0.274, *P* < 0.05). Univariate logistic regression analysis displayed that age (OR = 0.938; *P*=0.043), postprandial glucose/C-peptide (OR = 0.851; *p* ≤ 0.001), insulin resistance index (OR = 0.219; *p* ≤ 0.001), serum cystatin C (OR = 0.113; *p* ≤ 0.001), and uric acid (OR = 0.989; *P*=0.001) were risk factors for the risk of disease progression in patients with diabetic nephropathy. Multivariate logistic regression analysis exhibited that postprandial glucose/C-peptide (OR = 0.747; *P*=0.004), insulin resistance index (OR = 0.072; *P*=0.012), serum cystatin C (OR = 0.023; *P*=0.020), and uric acid (OR = 0.967; *P*=0.039) were independent risk factors for the risk of disease progression in patients with diabetic nephropathy. The ROC curve results demonstrated that the AUC of postprandial glucose/C-peptide predicting the risk of disease progression in patients with diabetic nephropathy was 0.931. Postprandial glucose/C-peptide, insulin resistance index, serum cystatin C, and uric acid are correlated with 24hUAER and eGFR. Postprandial glucose/C-peptide, insulin resistance index, serum cystatin C, and uric acid are independent risk factors for the risk of disease progression in patients with diabetic nephropathy. Among them, postprandial glucose/C-peptide can be employed as a crucial indicator to predict the risk of disease progression in diabetic nephropathy patients.

## 1. Introduction

Diabetic nephropathy is a rapidly progressive disease and has no obvious clinical symptoms in the early stage. Renal function damage has occurred at the time of diagnosis. Most patients may suffer from end-stage renal disease in a relatively short period, and ultimately, renal replacement therapy is required to maintain their lives [1, 2]. Therefore, it is a huge clinical challenge to identify the risk of diabetic nephropathy progression early and to timely intervene for delaying the progression of diabetic nephropathy. The latest study has found that serum C-peptide is a secretory product of islet B cells. If islet B cells are damaged, serum C-peptide levels can decrease, which is helpful for the early diagnosis of type 2 diabetes [3]. Nevertheless, there are few studies addressing the correlation between C-peptide and the progression of diabetic nephropathy, and C-peptide alone has certain limitations. Taken together, this study sought to investigate the correlation between the glucose/C-peptide ratio and the risk of disease progression in diabetic nephropathy patients to provide a theoretical basis for the clinic.

## 2. Data and Methods

### 2.1. General Data

Ninety-three patients with diabetic nephropathy, who were treated in the Chun'an Branch of Zhejiang Provincial People's Hospital, China, between January 2016 and January 2019, were enrolled in this study as subjects. In accordance with the disease progression, the patients were assigned to a progression group (*n* = 59) and a nonprogression group (*n* = 34).

### 2.2. Inclusion and Exclusion Criteria

Inclusion criteria are as follows: (1) accordance with the diagnostic criteria for diabetic nephropathy in Expert Consensus on the Prevention and Treatment of Diabetic Nephropathy (2014 edition), formulated by Chinese Medical Association Diabetes Branch [4]; (2) age range from 18 to 75 years; and (3) good compliance. Exclusion criteria are as follows: (1) kidney disease induced by other causes; (2) severe organic diseases, such as heart, lung, liver, brain, and kidney; (3) taking nephrotoxic drugs within the past one month; (4) combination with severe infection; (5) CKD stage 5 or receiving renal replacement therapy; (6) combination with malignant tumors; (7) lactating or pregnant women; and (8) incomplete clinical data.

### 2.3. Methods

All patients were treated in accordance with *Expert Consensus on the Prevention and Treatment of Diabetic Nephropathy* (2014 Edition) [4], mainly to reasonably control blood glucose (choosing oral hypoglycemic drugs or insulin injections in accordance with blood glucose level to control blood glucose to an average level), control blood pressure (choosing angiotensin-converting enzyme inhibitor or angiotensin II receptor antagonist treatment in accordance with the conditions of the patient to control blood pressure to a normal range), and control blood lipids (applying statin drug therapy to control blood lipids to a normal range). Simultaneously, patients were given health education to cultivate healthy living habits (low-glucose, low-salt, and low-fat diet combined with appropriate exercise training).

### 2.4. Indicator Detection

5 ml of venous blood was collected from all patients in the early morning, placed at room temperature for 30 minutes, and centrifuged at 3000 r/min for 15 minutes in a centrifuge. The supernatant was taken for testing: (1) fasting blood glucose, glycosylated hemoglobin (HbA1c), high-density lipoprotein cholesterol (HDL-C), low-density lipoprotein cholesterol (LDL-C), triglycerides (TG), total cholesterol (TC), blood urea nitrogen (BUN), and serum creatinine (SCr) were detected by a Beckman Coulte automatic biochemical analyzer. (2) C-peptide was examined by an automatic chemiluminescence immunoassay analyzer (DPC, USA). (3) 24 hUAER was detected by an IMMULITE automatic chemiluminescence immunoassay analyzer. The diagnostic criterion for the progression of diabetic nephropathy is that the glomerular filtration rate drops by 30% within 24 months.

### 2.5. Statistical Methods

All data are processed using SPSS 22.0. The count data were expressed as a rate (%) and compared with the *χ*^2^ test. The measurement data were expressed as the mean ± standard deviation $\left(\bar{\chi }\pm s\right)$, and the *t*-test was used for comparison. Spearman's correlation analysis was performed between the two variables. Logistic regression was utilized to analyze the independent risk factors for the risk of disease progression in diabetic nephropathy patients. A value of *P* < 0.05 was considered statistically significant.

## 3. Results

### 3.1. Comparison of Clinical Data between the Progression and Nonprogression Groups

There was no significant difference in sex, BMI, smoking, duration of diabetes, blood pressure, BUN, SCr, TG, TC, HDL-C, and LDL-C between the progression and nonprogression groups (*P* > 0.05). The differences in age, glucose/C-peptide, glycosylated hemoglobin, insulin resistance index, serum cystatin C, uric acid, 24 hUAER, and eGFR were significantly different between the progression and nonprogression groups (*P* < 0.05).  Table 1 shows the comparison of clinical data between the progression and nonprogression groups.

### 3.2. Correlation of Age, Glucose/C-Peptide, Glycosylated Hemoglobin, Insulin Resistance Index, Serum Cystatin C, and Uric Acid with 24hUAER and eGFR

Pearson's linear correlation analysis displayed that glucose/C-peptide, insulin resistance index, serum cystatin C, and uric acid were positively correlated with 24hUAER (*r* = 0.514, 0.345, 0.311, 0.279, *P* < 0.05). Age, glucose/C-peptide, insulin resistance index, serum cystatin C, and uric acid were negatively correlated with eGFR (*r* = −0.210, −0.610, −0.351, −0.347, −0.274, *P* < 0.05).  Table 2 shows the correlation of age, glucose/C-peptide, glycosylated hemoglobin, insulin resistance index, serum cystatin C, and uric acid with 24 hUAER and eGFR.

### 3.3. Univariate Logistic Regression Analysis of Risk Factors Related to the Risk of Disease Progression in Diabetic Nephropathy Patients

Univariate logistic regression analysis exhibited that age (OR = 0.938; *P*=0.043), postprandial glucose/C-peptide (OR = 0.851; *p* ≤ 0.001), insulin resistance index (OR = 0.219; *p* ≤ 0.001), serum cystatin C (OR = 0.113; *p* ≤ 0.001), and uric acid (OR = 0.989; *P*=0.001) were risk factors for the risk of disease progression in diabetic nephropathy patients.  Table 3 shows the univariate logistic regression analysis of risk factors related to disease progression in patients with diabetic nephropathy.

### 3.4. Multivariate Logistic Regression Analysis of Risk Factors Related to the Risk of Disease Progression in Diabetic Nephropathy Patients

Multivariate logistic regression analysis demonstrated that postprandial glucose/C-peptide (OR = 0.747; *P*=0.004), insulin resistance index (OR = 0.072; *P*=0.012), serum cystatin C (OR = 0.023; *P*=0.020), and uric acid (OR = 0.967; *P*=0.039) were independent risk factors for the risk of disease progression in diabetic nephropathy patients.  Table 4 shows the multivariate logistic regression analysis of risk factors related to the risk of disease progression in diabetic nephropathy patients.

### 3.5. ROC Curve of Postprandial Glucose/C-Peptide Predicting the Risk of Disease Progression in Diabetic Nephropathy Patients

The AUC of postprandial glucose/C-peptide predicting the risk of disease progression was 0.931 in diabetic nephropathy patients (95% CI: 0.881–0.980, *p* ≤ 0.001); the cut-off value was 55.976; the sensitivity was 80%; the specificity was 94%.  Figure 1 shows the ROC curve of postprandial glucose/C-peptide predicting the risk of disease progression in diabetic nephropathy patients.

## 4. Discussion

Chronic hyperglycemia can damage the kidney and induce diabetic nephropathy, which is one of the severe complications and one of the main causes of death in diabetic patients [5]. The duration of the disease is long, and the kidney damage is relatively insidious. In the initial stage, the disease mainly presents the thickening of the glomerular basement membrane, accompanied by glomerular nodular, diffuse changes, or glass-like changes in the renal arterioles, which increases the resistance of the renal blood vessels and diminishes the renal blood flow. With the progression and gradual deterioration, end-stage renal disease eventually appeared and seriously affected the health of patients [6, 7]. C-peptide secreted by the pancreas can precisely reflect endogenous insulin secretion, thereby reflecting blood sugar levels [8, 9]. Nevertheless, it remains poorly understood whether C-peptide is associated with diabetic nephropathy and whether C-peptide objectively and accurately reflects the progression of diabetic nephropathy. Taken together, this study mainly investigated the correlation between the glucose/C-peptide ratio and the risk of disease progression in diabetic nephropathy patients to provide theoretical guidance for the clinic.

This study confirmed that postprandial glucose/C-peptide, insulin resistance index, serum cystatin C, and uric acid were positively correlated with 24 hUAER. Age, postprandial glucose/C-peptide, insulin resistance index, serum cystatin C, and uric acid were negatively correlated with eGFR. Blood biochemical examination is one of the main methods in the diagnosis and treatment of diabetes. It can effectively diagnose diseases and understand the development of diseases. The reason is that C-peptide, mainly secreted by islet *β* cells, is relatively stable in the body and is not interfered by other factors, cannot be cleared by the liver, or be interfered by exogenous insulin, and can reflect the function of islet cells. The C-peptide level cannot only reflect the endogenous insulin level but cannot objectively reflect blood glucose level [10, 11]. The increase in postprandial glucose/C-peptide level can precisely reflect the hyperglycemia state. High blood sugar levels can increase the burden on the kidney and damage the kidney [12]. Thus, the postprandial glucose/C-peptide is correlated with 24 hUAER and eGFR. Insulin resistance can reduce the sensitivity of cells to insulin in the body, increase blood glucose, trigger a series of cell signal cascades, and cause glomerular epithelial cells, mesangial cells, and podocytes to produce chemokines and growth factors, thereby causing damage to the renal basement membrane and tubules, and proteinuria [13, 14]. Therefore, the insulin resistance index is correlated with 24 hUAER and eGFR. Serum cystatin C is a small molecule protein, and its production rate is not affected by age, inflammation, or medicines. Serum cystatin C is relatively constant, can almost be filtered from the glomerulus, is completely reabsorbed, and degraded by renal tubular epithelial cells, but cannot return to the blood [15, 16]. Renal tubular epithelial cells do not secrete serum cystatin C into the lumen [17, 18]. If the glomerular filtration function is slightly damaged, the serum cystatin C can continue to increase, so serum cystatin C is correlated with 24 hUAER and eGFR. Uric acid, the final product of human purine metabolism, is mainly excreted from the body through the kidney and intestine. Under normal circumstances, the amount of uric acid ingested and excreted by the human body is dynamic equilibrium [19]. As for abnormal renal function, the increased uric acid level can further inhibit the bioavailability of endothelial nitric oxide synthase, thereby damaging the vascular endothelial cells of the kidney and aggravating kidney damage [20, 21]. Therefore, uric acid is correlated with 24 hUAER and eGFR.

Univariate logistic regression model analysis results verified that age, postprandial glucose/C-peptide, insulin resistance index, serum cystatin C, and uric acid were correlated with the risk of disease progression in diabetic nephropathy patients. Multivariate logistic regression model analysis results concluded that postprandial glucose/C-peptide, insulin resistance index, serum cystatin, and uric acid were independent risk factors for the risk of disease progression in patients with diabetic nephropathy, indicating that postprandial glucose/C-peptide, insulin resistance index, serum cystatin C, and uric acid can affect the risk of disease progression in patients with diabetic nephropathy to a certain extent. Proinsulin is the precursor of insulin, which is decomposed into three parts under the action of enzymes. The front and rear segments are reconnected to become insulin. The middle segment is serum C-peptide, which has an equimolecular relationship with insulin. Serum C-peptide is not inactivated by liver enzymes, and its half-life is 10-11 min, which is longer than that of insulin by 4.8 min. Therefore, the function of islet B cells is more valuable to evaluate by the level of serum C-peptide. In addition, exogenous insulin does not contain C-peptide, and the serum C-peptide level of patients undergoing insulin treatment can still reflect the function of islet B cells. Therefore, the evaluation of the effect of postprandial blood glucose/C peptide on diabetes can better reflect the reserve function of islet B cells. Insulin resistance is one of the pathogenesis of type 2 diabetes. Insulin resistance is positively correlated with urinary microalbumin in diabetic patients. Hyperuricemia is one of the most important risk factors for early diabetic nephropathy. The level of serum uric acid is closely related to glucose metabolism. The serum uric acid level in patients with newly diagnosed type 2 diabetes decreases with the increase of fasting blood glucose, which may be related to increased diuresis, increased urine output, and increased excretion of blood uric acid.

The ROC curve was utilized to assess the predictive value of postprandial glucose/C-peptide on the risk of disease progression in patients with diabetic nephropathy. The results showed that the AUC of postprandial glucose/C-peptide was 0.931, suggesting that postprandial glucose/C-peptide can be applied as an important indicator to predict the risk of disease progression in patients with diabetic nephropathy. The results from the present study are consistent with those of Jone et al. [22]. The level of glycosylated hemoglobin is positively correlated with the concentration of blood glucose, which is an irreversible reaction, which is related to the degree of poor disease control and has significant diagnostic significance. Glycosylated hemoglobin (HbA1c) is a medium and long-term index reflecting the level of glucose in the blood. The blood sugar level in 30 d has a 50% effect on it, while 90–120 d only affects 10%. It has become the golden standard for observing the control of diabetes. The C peptide is one of the end products of proinsulin cleavage. Due to its slow clearance, it is not affected by liver enzyme inactivation, and can better reflect the pancreas *β* cells. The ability of cells to produce and secrete insulin can be used to guide clinical medication.

Simultaneously, this study still has limitations. The glucose/C-peptide ratio is an average result over a period of time and does not represent a single time point, so it cannot be compared with such results. In addition, the relatively small sample size and relatively single source can impact the research results. Thus, we will conduct a large-sample, multicenter, and different time-point investigation in the future.

## 5. Conclusion

In summary, postprandial glucose/C-peptide, insulin resistance index, serum cystatin C, and uric acid are correlated with 24 hUAER and eGFR. Postprandial glucose/C-peptide, insulin resistance index, serum cystatin C, and uric acid are independent risk factors for the risk of disease progression in patients with diabetic nephropathy. Among them, postprandial glucose/C-peptide can be employed as a crucial indicator to predict the risk of disease progression in diabetic nephropathy patients.

## Figures and Tables

**Figure 1:** ROC curve of postprandial glucose/C-peptide predicting the risk of disease progression in diabetic nephropathy patients.

**Table 1:** Comparison of clinical data between the progression and nonprogression groups.

Clinical data		Progression group (*n* = 59)	Nonprogression group (*n* = 34)	Statistics	*P*
Age (years)		61.36 ± 7.38	58.10 ± 6.95	2.098	0.039
Sex (*n*(%))	Female	33(55.93)	22(64.71)	0.687	0.407
	Male	26(44.07)	12(35.29)		
BMI (kg/m^2^)		25.33 ± 3.42	24.16 ± 3.09	1.645	0.104
Smoking (*n*(%))		42(71.19)	24(70.59)	0.004	0.951
Duration of diabetes (years)		11.54 ± 1.78	10.86 ± 1.54	1.861	0.066
SBP (mmHg)		136.73 ± 10.92	133.68 ± 10.46	1.317	0.191
DBP (mmHg)		75.24 ± 12.66	73.38 ± 11.59	0.703	0.484
Glucose/C-peptide		76.05 ± 22.05	42.91 ± 9.72	8.295	≤0.001
Glycosylated hemoglobin (%)		9.51 ± 2.01	8.50 ± 2.84	2.000	0.048
Insulin resistance index		3.78 ± 0.81	2.84 ± 0.77	5.495	≤0.001
Serum cystatin C (mg/l)		2.43 ± 0.71	1.86 ± 0.22	4.512	≤0.001
Uric acid (*μ*mol/l)		343.80 ± 77.51	289.56 ± 55.98	3.575	0.001
BUN (mmol/l)		8.47 ± 2.82	8.16 ± 2.25	0.548	0.585
SCr (*μ*mol/l)		75.38 ± 23.64	72.96 ± 21.73	0.489	0.626
TG (mmol/l)		2.20 ± 0.75	2.13 ± 0.82	0.419	0.676
TC (mmol/l)		4.53 ± 1.21	4.42 ± 1.18	0.426	0.671
HDL-C (mmol/l)		1.41 ± 0.35	1.52 ± 0.48	-1.271	0.207
LDL-C (mmol/l)		3.27 ± 0.81	3.15 ± 0.76	0.703	0.484
24 hUAER (*μ*g/min)		614.09 ± 102.13	347.13 ± 81.14	13.044	≤0.001
eGFR (ml/(min.1.73 m^2^)		37.64 ± 12.20	69.77 ± 10.57	-12.828	≤0.001

**Table 2:** Correlation of age, glucose/C-peptide, glycosylated hemoglobin, insulin resistance index, serum cystatin C, and uric acid with 24 hUAER and eGFR.

Item	24 hUAER		eGFR	
	*r*	*P*	*r*	*P*
Age	0.084	0.425	−0.210	0.044
Glucose/C-peptide	0.514	≤0.001	−0.610	≤0.001
Glycosylated hemoglobin	0.185	0.076	−0.068	0.520
Insulin resistance index	0.345	0.001	−0.351	0.001
Serum cystatin C	0.311	0.002	−0.347	0.001
Uric acid	0.279	0.007	−0.274	0.008

**Table 3:** Univariate logistic regression analysis of risk factors related to disease progression in patients with diabetic nephropathy.

Factor	*B*	Standard error	Wals	*P*	OR	95% CI	
						Lower limit	Upper limit
Age	−0.064	0.032	4.088	0.043	0.938	0.882	0.998
Postprandial glucose/C-peptide	−0.162	0.036	19.987	≤0.001	0.851	0.792	0.913
Glycosylated hemoglobin	−0.182	0.094	3.779	0.052	0.833	0.693	1.001
Insulin resistance index	−1.521	0.358	18.027	≤0.001	0.219	0.108	0.441
Serum cystatin C	−2.184	0.601	13.210	≤0.001	0.113	0.035	0.366
Uric acid	−0.011	0.004	10.090	0.001	0.989	0.982	0.996

**Table 4:** Multivariate logistic regression analysis of risk factors related to the risk of disease progression in diabetic nephropathy patients.

Factor	*B*	Standard error	Wals	*P*	OR	95% CI	
						Lower limit	Upper limit
Age	0.109	0.111	0.966	0.326	1.115	0.897	1.385
Postprandial glucose/C-peptide	−0.291	0.102	8.211	0.004	0.747	0.613	0.912
Insulin resistance index	−2.637	1.050	6.306	0.012	0.072	0.009	0.561
Serum cystatin C	−3.778	1.623	5.418	0.020	0.023	0.001	0.551
Uric acid	−0.034	0.016	4.282	0.039	0.967	0.937	0.998

## Data Availability

The data availability of this study fully met the requirements of the journal. The original information is available through the corresponding author.
